# Study on the Application of Doxorubicin-Loaded Magnetic Nanodrugs in Targeted Therapy of Liver Cancer

**DOI:** 10.1155/2022/2756459

**Published:** 2022-02-22

**Authors:** Lei Wang, Liping Liang, Shuzhen Shi, Chao Wang

**Affiliations:** ^1^Department of Pharmacy, Qingdao Jiaozhou Central Hospital, Qingdao, 266300 Shandong, China; ^2^Pharmacy Department of Qingdao Chest Hospital, Qingdao, 266043 Shandong, China

## Abstract

Doxorubicin (DOX) has been widely recognized as effective in anticancer therapy; however, the additional organ toxicity and low targeting of DOX in antitumor activity remains unaddressed. The aim of this study was to use the drug carrier dextran/polylactic acid (DEX/PLA) and paramagnetic Fe3O4 to improve the targeting of DOX in liver cancer treatment while reducing its potential organ toxicity. Our experimental results show that the combination drug (Fe3O4@DEX/PLA-DOX) exhibits strong hepatocarcinogenic inhibition and low cytotoxicity and that this modified drug provides a better option for clinical liver cancer treatment.

## 1. Introduction

Liver cancer is one of the six common cancers in the world. It can be divided into primary liver cancer and secondary liver cancer. Primary liver cancer refers to the primary tumor of the liver, and secondary liver cancer refers to other parts of the liver. The tumor has metastasized to the tumor in the liver [1–4]. The incidence of liver cancer is extremely high, and it is also the fourth leading cause of cancer deaths. And the survey shows that the incidence of liver cancer is higher in underdeveloped areas. East Asia, South Asia, and North Asia are all high-risk areas for liver cancer [5]. The causes of liver cancer are still unclear. Alcoholism, obesity, cirrhosis, hepatitis B, hepatitis C, fatty liver, and diabetes are all risk factors for liver cancer [6, 7]. In terms of treatment, liver resection and liver transplantation have always been the first choice for the treatment of liver cancer [8, 9]. In addition, chemotherapy, radiotherapy, molecular targeted therapy, immunotherapy, antiviral therapy, traditional Chinese medicine, and other adjuvant sexual therapy can effectively inhibit liver cancer. Among them, radiotherapy is not a first-line treatment plan for liver cancer, but it can be used as an effective means for local treatment of liver cancer [10–12]. Chemotherapy is a common treatment method in traditional cancer treatment, but it is more harmful to the liver, and it is easy to aggravate the symptoms of liver cirrhosis and hepatitis. It is currently commonly used in the treatment of advanced liver cancer [13]. Antiviral therapy mainly targets liver cancer caused by hepatitis B and C. At the same time, it can also inhibit the replication of the hepatitis virus caused by Feilaozi-targeted drugs and chemotherapy drugs. It can be used throughout the treatment of liver cancer [14–16]. Immunotherapy can enhance the body's own immune function, break immune tolerance, and stimulate the body's tumor-specific immunity to delay tumor development [17]. Molecular targeted therapy has now occupied an important position in the treatment of liver cancer. Compared with other therapeutic drugs, it has low toxicity and high selectivity. It can target the disease through a variety of signaling pathways, which is the focus of current research [18–20]. In addition, traditional Chinese medicine for the treatment of liver cancer is gradually being recognized by the public, and studies have shown that it can effectively inhibit the recurrence and metastasis of liver cancer.

Doxorubicin (DOX), as an anthracycline antibiotic, can be trimerized between DNA base pairs, triggering topoisomerase II to cleave DNA, thereby causing damage to the tertiary structure of DNA [21]. In addition, as a cell cycle nonspecific drug, it can cause cytotoxic effects on the cells at various stages, so it is widely used in the treatment of breast cancer, lung cancer, liver cancer, ovarian cancer, bladder cancer, and other cancers. However, DOX usually causes high fever, nausea, vomiting, phlebitis, bone marrow transplantation, and severe cardiotoxicity [22]. Therefore, how to reduce the occurrence of side effects plays an important role in clinical applications. Targeted nanoformulation is a drug formulation that can identify specific targets of the lesion and can be targeted for delivery. It can usually be delivered by carriers such as liposomal microspheres, microcapsules, and nanoparticles. It can improve the problem of poor solubility of drugs and at the same time reduce the damage of drugs to other parts except for the lesion [23]. Magnetic nanoparticles can achieve targeted drug delivery for liver cancer by loading drugs on carriers containing magnetic materials. Common magnetic targeting materials include ferrite magnetic materials, Fe3O4 iron powder, and magnetic alloy materials [24].

Dextran (DEX) is a water-soluble polysaccharide with a linear backbone, which has good biocompatibility and nontoxic effects. In addition, DEX has good reactivity, can load a variety of biologically active molecules, and has good excipient characteristics when used in the modification of magnetic nanoparticles, which can effectively promote application research in tumors and immunodetection [25]. Polylactic acid (PLA) is a bio-based renewable and degradable material with a wide range of sources. It is widely used in packaging materials, fibers, clothing, construction, agriculture, and medical and health fields. It is a good drug carrier material [26]. Based on this, this study used DOX as a therapeutic drug and DEX/PLA as a drug carrier, modified with Fe3O4 to obtain Fe3O4@DEX/PLA-DOX and study its inhibitory effect on liver cancer.

## 2. Materials and Methods

### 2.1. Reagent

Ferrous sulfate (FeSO_4_∙4H_2_O), iron chloride (FeCl_3_∙6H_2_O), ammonia, N-N′-dicyclohexylcarbodiimide, 4-dimethylaminopyridine, acetone, dichloromethane, and 3-(4,5-Dimethylthiazol-2-yl)-2,5-diphenyltetrazolium bromide were purchased from Shanghai Yien Chemical Technology Co., Ltd. (Shanghai, China). PLA and DEX were provided by Nanjing Dulai Biotechnology Co., Ltd. (Jiangsu, China). Fetal bovine serum, DMEM medium, and DMSO were purchased from Hangzhou Jiangbin Biotechnology Co., Ltd. (Zhejiang, China).

### 2.2. Instrument

The Shimadzu high-performance liquid chromatograph Essentia LC-15C (HPLC) used to detect the content of DOX was purchased from Shimadzu Corporation (Kyoto, Japan). The XH-EC-8850 conductivity detector is manufactured by Beijing Heng Aode Instrument Co., Ltd. (Beijing, China). The 120 kV transmission electron microscope HT7800 was purchased from Hitachi Limited (Tokyo, Japan). The micro high-speed refrigerated centrifuge C1650R-230V was purchased from Beijing Lept Scientific Instrument Co., Ltd. (Beijing, China). Zhejiang Aosheng FlexA-200 full-wavelength enzyme label analyzer was provided by Hangzhou Aosheng Instrument Co., Ltd. (Zhejiang, China).

Mouse hepatocellular carcinoma cells (H22 cells) were provided by Wuhan Punuosai Life Technology Co., Ltd. (Hubei, China). BABL/c mice were purchased from Nanjing Junke Biological Engineering Co., Ltd. (Jiangsu, China). All animal-related experimental operations involved in this experiment comply with international ethical standards.

### 2.3. Preparation and Characterization of Fe_3_O_4_@DEX/PLA-DOX

#### 2.3.1. Preparation of Magnetic Nanoparticles

0.75 g of FeSO_4_∙4H_2_O and 1.5 g of FeCl_3_∙6H_2_O were stirred in 50 mL of double-distilled water, adjusted to pH = 9.5 with NH_3_∙H_2_O, and then washed until the conductivity was lower than 50 *μ*s to obtain Fe_3_O_4_ nanoparticles. Disperse Fe_3_O_4_ nanoparticles in 50 mL of double distilled water using an ultrasonic cleaner to obtain Fe_3_O_4_ magnetic nanoparticles solution.

#### 2.3.2. Preparation of DEX/PLA Vector

500 mg of PLA, 200 mg of N-N′-dicyclohexylcarbodiimide, and 15 mg of 4-dimethylaminopyridine were placed in the flask, 30 mL of DMSO was added, and the mixture was stirred and dissolved at 60°C. Continue the reaction for 30 min. Immediately add 250 mg of DEX, and react for two days under nitrogen protection. The reaction mixture was put into a dialysis bag and dialyzed in running water for 48 h. The suspension was centrifuged at 12,000 rpm for 20 min, the supernatant was lyophilized and dissolved in acetone solution for washing, and the solid lyophilized was obtained by suction filtration to prepare the DEX/PLA carrier.

#### 2.3.3. Preparation of Fe_3_O_4_@DEX/PLA-DOX

Fe_3_SO_4_ magnetic nanoparticles were dissolved in DMSO, added DEX/PLA carrier, stirred uniformly at 60°C, and reacted for 24 h. When the reaction was over, put them in a dialysis bag and dialyze with double-distilled water for 48 h. Centrifuge the suspension in the dialysis bag at 3,000 rpm for 10 min. The supernatant was lyophilized and dissolved in an acetone solution. The solid after suction filtration was washed and then lyophilized to obtain Fe_3_O_4_@DEX/PLA graft things.

The preparation of Fe_3_O_4_@DEX/PLA-DOX adopts the solvent diffusion method. Dissolve DOX in double-distilled water and add it to Fe_3_O_4_@DEX/PLA graft solution in DMSO at a ratio of 1 : 20, and transfer it to dialysis. The inside of the bag was dialyzed with double-distilled water for 20 h in the dark and then centrifuged at 3,000 rpm for 10 min. The supernatant was collected to obtain the Fe_3_O_4_@DEX/PLA-DOX solution. Use electron microscopy to characterize and measure its particle size at the same time.

### 2.4. Encapsulation Rate and Drug Loading Rate Determination

Dissolve Fe_3_O_4_@DEX/PLA-DOX in 5.0 mL of dichloromethane, add 10 mL of PBS solution after it is completely dissolved, mix well and refine for 2.0 h, separate and collect the water phase, add 5.0 mL of PBS solution again to the oil phase, mix well and then stand for layering, collect the aqueous phase, combine the two collected aqueous phases, dilute 10 times and centrifuge at 3,000 rpm for 10 min, take the supernatant, and use HPLC to detect the supernatant. The content of DOX in the liquid is calculated, and its encapsulation rate and drug loading rate are calculated.

### 2.5. *In Vitro* Release Capacity Determination

Take Fe_3_O_4_@DEX/PLA-DOX powder and place it in a dialysis bag (DOX as a control group), and use PBS solution for dialysis treatment. To simulate the internal environment, the pH is set to three gradients of 4.0, 6.28, and 7.4, and set the dialysis environment to a constant temperature environment of 37°C, and take out 3.0 mL of dialysate at 0, 0.5, 1.0, 2.0, 4.0, 6.0, 12, 24, 48, 72, 96, and 120 h, and replenish it. Use HPLC to detect the amount of drug released at each time point.

### 2.6. *In Vitro* Toxicity Determination

The *in vitro* toxicity of Fe_3_O_4_@DEX/PLA-DOX nanomedicine was studied in H22 cells. Use DMEM medium containing 10% fetal bovine serum and culture to logarithmic phase at 37°C and 5.0% CO_2_, and use MTT for detection. In the whole experiment, DOX was used as the control group, Fe_3_O_4_@DEX/PLA blank carrier was used as the blank group, and Fe_3_O_4_@DEX/PLA-DOX was used as the experimental group. The MTT solution was added after cocultivation with cells for 0, 24, 48, and 72 h. After incubation for 4.0 h, discard the MTT solution, add DMSO for color development, and detect the absorbance at 570 nm in the microplate reader.

### 2.7. Analysis of the Effect of Inhibiting Liver Cancer *In Vivo*

#### 2.7.1. Construction of Liver Cancer Model

The hepatocarcinoma model was constructed by tumor cell heterotopic inoculation. H22 cells in the logarithmic growth phase were diluted to a cell suspension with a concentration of 1.0 × 10^7^ cells/mL and inoculated into the right scapula of SPF BABL/c mice. They were reared subcutaneously and normally (the control group was not vaccinated), and the diameter of the tumor of the mice was recorded with cursor cardboard every day, and the administration was started when the diameter reached about 0.5 cm.

#### 2.7.2. Treatment Programs

The mice were randomly divided into the control group, model group, DOX group, and Fe_3_O_4_@DEX/PLA-DOX group. Each group had 12 mice. Except for the control group and model group, the DOX group and Fe_3_O_4_@ were injected with normal saline through the tail vein. The DEX/PLA-DOX group was given the same amount of DOX and Fe_3_O_4_@DEX/PLA-DOX, once every 5 days for a total of 3 doses. On the 21st day after the administration, 6 mice in each group were sacrificed. The tumor is removed and weighed. The remaining mice were fed naturally to death, and their average survival time was observed. Its therapeutic mechanism for liver cancer is shown in Figure 1.

### 2.8. Targeting Effect

The blood, heart, liver, kidney, and tumor tissues of the sacrificed mice were frozen and ground, added with saline, mixed well, and centrifuged at 12,000 rpm for 20 min. The supernatant was used to detect the main tissues in the HPLC content of DOX.

## 3. Results and Discussion

### 3.1. Fe_3_O_4_@DOX-DEX/PLA Morphology Characteristics

Fe_3_O_4_@DEX/PLA-DOX nanoparticles were characterized by electron microscopy, and the characterization results are shown in Figure 2. Its appearance is spherical, with an average particle size of 86.31 ± 10.68 nm. Because its particle size is less than 100 nm, it has high permeability and can freely enter and exit the tumor site with a multivascular structure, which is beneficial to the treatment of cancer.

### 3.2. Encapsulation Rate and Drug Loading Rate

Figure 3 shows the test results of the encapsulation rate and drug loading rate of Fe_3_O_4_@DEX/PLA-DOX nanoparticles. After testing, the encapsulation rate of Fe_3_O_4_@DEX/PLA-DOX nanoparticles is 59.45 ± 3.64%, and the drug loading rate is 24.69 ± 0.94%. It has good encapsulation and drug loading effects on DOX.

### 3.3. *In Vitro* Release Ability

In order to simulate the release of Fe_3_O_4_@DEX/PLA-DOX nanoparticles in the body, the simulated release was performed in solutions of different pH (Figure 4). By comparison, Fe_3_O_4_@DEX/PLA-DOX nanoparticles were released rapidly within the first 24 h, and the subsequent release was slow. And compared with the released results of DOX, it proves that Fe_3_O_4_@DEX/PLA-DOX nanoparticles have a slow release effect. At the same time, the comparison of the release effect at different pH shows that Fe_3_O_4_@DEX/PLA-DOX nanoparticles have a better release effect in acidic media. Because the cancer tissue and its surrounding environment are usually acidic, it can accurately reach the cancer tissue and inhibit it.

### 3.4. *In Vitro* Toxicity Determination

Taking H22 cells as the research object, the inhibitory effect of Fe_3_O_4_@DEX/PLA-DOX nanoparticles on cell proliferation was studied (Figure 5). It was found that the DEX/PLA vector had almost no inhibitory effect on the cells, which indicated that the DEX/PLA vector had no toxic effect on the west. Fe_3_O_4_@DEX/PLA-DOX nanoparticles have obvious toxic effects on H22 cells. The cell proliferation rate at 72 h is only 43.65 ± 10.29%. Compared with the DOX group, its inhibitory effect on H22 cells is more obvious. This result proves that Fe_3_O_4_@DEX/PLA-DOX nano has a stronger inhibitory effect on liver cancer.

### 3.5. Ability to Inhibit Liver Cancer *In Vivo*

Animal experiments are used to simulate the *in vivo* inhibitory ability of Fe_3_O_4_@DEX/PLA-DOX nanoparticles on liver cancer.  Figure 6(a) shows the effect of Fe_3_O_4_@DEX/PLA-DOX on the weight of mouse liver cancer tumors. Compared with the model group, the tumor body of the Fe_3_O_4_@DEX/PLA-DOX group was significantly reduced. After 21 days of the administration, the tumor weight decreased to 213.62 ± 42.65 mg, while the tumor weight of the mice in the DOX group was 438.47 ± 53.42 mg; this result further proves that Fe_3_O_4_@DEX/PLA-DOX nanoparticles are better than DOX in inhibiting liver cancer. At the same time, the survival time results of each group of mice in Figure 6(b) show that the mice in the Fe_3_O_4_@DEX/PLA-DOX group have a longer survival time, reaching 63 days of action, while the DOX group is only 36 days. It proves that Fe_3_O_4_@DEX/PLA-DOX nanoparticles can effectively prolong the survival time of mice with liver cancer.

### 3.6. Targeting

In order to investigate the targeting of Fe_3_O_4_@DEX/PLA-DOX to liver cancer, the DOX content in the main organs of mice in the Fe_3_O_4_@DEX/PLA-DOX group and the DOX group was detected (Figure 7). The results showed that the Fe_3_O_4_@DEX/PLA-DOX content in the tumor was up to 7.31 ± 1.02 *μ*g/g, while the DOX group was only 2.53 ± 0.27 *μ*g/g. This proves that Fe_3_O_4_@DEX/PLA-DOX nanoparticles are targeted for liver cancer. In addition, since the DOX content in other main organs of mice in the Fe_3_O_4_@DEX/PLA-DOX group is lower, it can effectively avoid other organ damage caused by DOX.

## 4. Discussion

As an antibacterial and cytostatic drug, DOX is widely used in the treatment of malignant tumors [27]. Its targeted preparation can improve the inhibitory effect on tumors and reduce the toxic effect of DOX on nonfocal sites. It is a promising new way of administration [28]. With the increasing incidence of liver cancer, DOX targeting agents have also become a hot spot in current research [29, 30]. The ideal targeted preparation for inhibiting liver cancer can concentrate all the drugs on the lesion, but the current research is still unable to meet the standard. It can only relatively increase the distribution rate of DOX at the tumor site. Therefore, a new target or new type of action is sought. The carrier is the focus of current research.

Based on this, this work uses DOX as a therapeutic drug and DEX/PLA as a drug carrier, modified with Fe_3_O_4_ to obtain Fe_3_O_4_@DEX/PLA-DOX magnetic nanoparticles. The characterization results showed that Fe_3_O_4_@DEX/PLA-DOX nanoparticles were characterized, and the characterization results showed that Fe_3_O_4_@DEX/PLA-DOX has a spherical appearance and an average particle size of less than 100 nm. It has high permeability and can be used in the tumor site with a multivascular structure that can enter and exit freely, which is conducive to the treatment of cancer. Meanwhile, the encapsulation rate, drug loading rate, and in vitro drug release experiment results proved that it can effectively coat DOX and accelerate its release under acidic conditions to effectively inhibit cancer tissues. In vitro toxicity experiments proved that the carrier of Fe_3_O_4_@DEX/PLA-DOX is not cytotoxic and has good biological safety. Compared with DOX, Fe_3_O_4_@DEX/PLA-DOX has a better inhibitory effect on liver cancer. The results of in vivo experiments once again proved that Fe_3_O_4_@DEX/PLA-DOX can inhibit the growth of liver cancer and improve the survival time of liver cancer mice. In addition, compared with DOX, Fe_3_O_4_@DEX/PLA-DOX has stronger targeting of liver cancer tissue and can be used in the targeted therapy of liver cancer.

## 5. Conclusion

In this work, Fe3O4@DEX/PLA-DOX magnetic nanoparticles were prepared by using DEX/PLA as the drug carrier and modifying DOX with Fe3O4. The results of the in vivo and ex vivo experiments on structural characterization, encapsulation rate, drug loading rate, drug release capacity, toxicity, targeting, and ability to inhibit hepatocellular carcinoma found that Fe3O4@DEX/PLA-DOX has certain targeted inhibitory effect on hepatocellular carcinoma, and its inhibitory effect on hepatocellular carcinoma is stronger compared with that of DOX alone. The findings of this study are expected to provide a new way for the clinical treatment of liver cancer.

## Figures and Tables

**Figure 1:** The mechanism of action of doxorubicin-loaded magnetic nanomedicine (Fe_3_O_4_@DEX/PLA-DOX) on liver cancer.

**Figure 2:** Morphology characterization of magnetic nanomedicine containing doxorubicin (Fe_3_O_4_@DEX/PLA-DOX). (a) Electron microscopy characterization diagram. (b) Particle size.

**Figure 3:** Analysis of the encapsulation efficiency and drug loading rate of magnetic nanodrugs containing doxorubicin (Fe_3_O_4_@DEX/PLA-DOX).

**Figure 4:** Analysis of the drug release ability of doxorubicin-loaded magnetic nanodrugs (Fe_3_O_4_@DEX/PLA-DOX) at different pH. (a) pH = 4.00. (b) pH = 6.28. (c) pH = 7.40.

**Figure 5:** *In vitro* toxic effects of magnetic nanodrugs containing doxorubicin (Fe_3_O_4_@DEX/PLA-DOX) on H22 cells.

**Figure 6:** The inhibitory effect of doxorubicin-containing magnetic nanoparticles (Fe_3_O_4_@DEX/PLA-DOX) on liver cancer *in vivo*. (a) Tumor weight. (b) Survival time.

**Figure 7:** Targeting study of doxorubicin-containing magnetic nanoparticles (Fe_3_O_4_@DEX/PLA-DOX) on liver cancer.

## Data Availability

The data underlying the results presented in the study are available within the manuscript.
